The article "Variation in the Performance of MWCNT/ZnO Hybrid Material with pH for Efficient Antibacterial Agent" was published in 2022. Journal: Biomed Res Int.

# Variation in the Performance of MWCNT/ZnO Hybrid Material with pH for Efficient Antibacterial Agent

**DOI:** 10.1155/2022/1300157

**Published:** 2022-02-04

**Authors:** Saima Rafique, Shazia Bashir, Rizwan Akram, Farrukh Bashir Kiyani, Shagufta Raza, Mozaffar Hussain, Sayyeda Kaneez Fatima

**Affiliations:** ^1^Department of Physics, Air University, PAF Complex, E-9, Islamabad 44000, Pakistan; ^2^Department of Physics and Applied Mathematics, Pakistan Institute of Engineering and Applied Sciences, Islamabad 45650, Pakistan; ^3^Department of Microbiology, Quaid-i-Azam University, Islamabad, Pakistan

## Abstract

In the present work, multiwalled carbon nanotube (MWCNT)/zinc oxide (ZnO) nanoparticles at pH 6.0, 7.0, 8.0, and 10.0 were prepared through the coprecipitation method to improve the antibacterial activity. Morphological, structural, and optical analysis, such as Fourier transform infrared spectroscopy, X-ray diffraction, and field emission scanning electron microscopy, was used to investigate the formation of composites. Analysis revealed that there were variations in morphology from agglomerated structures to rod-like then flower-like structures as pH varied from 6.0 to 10.0. The MWCNT/ZnO composite enhanced the antibacterial activity especially for *Staphylococcus aureus* as a maximum 20 mm zone of inhibition was observed. The data presented in the present study proves that such composites are an efficient antibacterial agent and suitable for therapy for severe infections.

## 1. Introduction

The infectious disease affects human health and is caused by pathogenic microbes. For the treatment of these diseases, the first choice is antibiotics. However, high mutation and morphological changes lead to microbial resistance. To overcome this microbial resistance, a new nanoparticle-based strategy has gained more attention in recent times. Piktel et al. studied the antibacterial effect of various shape gold nanoparticles against different microbes [1]. Their study showed that gold nanoparticles can be used in combination to improve antimicrobial activity. Similarly, Qais et al. studied silver nanoparticles against Murraya koenigii (L.) and against multidrug-resistant pathogens [2]. The findings revealed that silver nanoparticles exhibit a wide range of activities against both gram-positive and gram-negative bacteria. Different types and shapes of nanoparticles have been used which are proposed as an alternative approach over traditional antibiotics to overcome bacterial resistance.

Zinc oxide has gained researcher's interest as it shows unique optical, chemical sensing, semiconducting, and piezoelectric properties due to its wide bandgap of 3.3 eV [3]. Besides, this zinc oxide and other metal oxides are widely used in biomedical applications [4]. Zinc oxide nanoparticles (ZnO NPs) are biosafe and act as a strong antibacteria for both gram-negative and gram-positive bacteria, and their antibacterial properties vary with the size of particles [5, 6]. Azam et al. performed a comparative study on antibacterial activity using three metal oxides such as zinc oxide (ZnO), copper oxide (CuO), and iron oxide (Fe_2_O_3_) [7]. They showed that ZnO nanoparticles showed excellent antimicrobial activity against both gram-positive and gram-negative bacteria as compared to CuO and Fe_2_O_3_. Similarly, Xie et al. have studied the antibacterial effect of zinc oxide (ZnO) nanoparticles on *Campylobacter jejuni* (*C. jejuni*) [8]. A remarkable effect of ZnO nanoparticles on antibacterial activity was obtained, and ZnO nanoparticles show a fatal effect against *C. jejuni*, even at low concentrations. Similarly, Rizwan et al. investigated the morphological variation such as sheet to microflowers by varying the pH of the solution [9]. However, Ribut et al. studied the morphological changes in ZnO NPs by the change of pH and how it affects their antibacterial properties [10]. They observed that the ZnO NPs synthesized at pH 11.0 act as the best antibacterial agent against *Escherichia coli* (*E. coli*). This suggests that ZnO nanoparticles act as a potential candidate for antibacterial activity and may have future applications to control the infection of a variety of bacterial strains.

Besides this, multiwalled carbon nanotubes (MWCNTs) show good electrical conductivity and chemical and thermal stability and also exhibit good antibacterial properties [11, 12]. The first reported literature for antibacterial activity of carbon nanotube (CNTs) was described by Kang et al., and they used single-wall carbon nanotubes as an antibacterial agent against *E. coli* [13]. Recently, the development of carbon nanotubes with metal/metal oxide nanoparticles has attracted much interest because of their large potential for technological applications [14]. David et al. reported the decoration of multiwalled carbon nanotubes (MWCNTs) with zinc oxide (ZnO), silver (Ag), and hydroxyapatite (HAp) nanoparticles to improve the antibacterial properties [15]. They conclude that antibacterial properties are enhanced using ZnO and Ag nanoparticles. Similarly, Upasani et al. reported the nanoribbon of zinc oxide (ZnO NR) and multiwalled carbon nanotube (MWCNT) composite film formation which exhibit a strong antimicrobial property [16]. Another antibacterial study on ZnO/MWCNT composites was performed by Sui et al. [17]. They evaluated that ZnO/MWCNTs act as an antimicrobial material and simultaneously, it is used for inactivating pathogenic bacteria. They showed that MWCNTs/ZnO exhibited strong antibacterial ability towards *E. coli*.

In this sequence, we have tried to explore the antibacterial activity of multiwalled carbon nanotubes (MWCNTs) and pH-based synthesized zinc oxide nanoparticles. In the present study, a novel nanocomposite, pH-based ZnO nanoparticles, and MWCNTs were expected to produce which is not reported yet that combine the properties of two functional materials to achieve more effective antibacterial properties, whereas *Staphylococcus aureus* (*S.A*), *Escherichia coli* (*E. coli*), *Klebsiella pneumoniae* (*K.P*), and *Pseudomonas aeruginosa* (*Pseudo*) bacteria were used to evaluate the antibacterial activity of the MWCNT/ZnO.

## 2. Experiment

### 2.1. Materials

The multiwalled carbon nanotube (MWCNT) with an average diameter of 18 ± 7 nm was purchased from Beijing DK Nano technology, China. Zinc chloride (ZnCl_2_), sodium hydroxide (NaOH), nitric acid (HNO_3_), and hydrochloric acid (HCl) were purchased from Sigma-Aldrich. All solutions used in experiments were prepared in deionized water.

### 2.2. Synthesis of Zinc Oxide Nanoparticles (ZnO NPs) at Different pH

Zinc oxide nanoparticles were synthesized by using the coprecipitation method [18]. Zinc chloride was dissolved in 100 ml of distilled water and continuously stirred at 80°C. While stirring is in process, concentrated sodium hydroxide was added to obtain different pH such as 6.0, 7.0, 8.0, and 10.0 as shown in Figure 1(a). After 2 hrs, white precipitates were formed which comprised zinc hydroxide and sodium chloride. Sodium chloride was separated from the solution by filtration. The filtered solution was dried in an oven for 4-6 hrs to obtain zinc oxide nanoparticles prepared at different pH in powdered form.

### 2.3. Functionalization of Multiwalled Carbon Nanotubes (MWCNTs)

For the functionalization of MWCNT, they were washed with 5 M HCl solution, wherein the functional group of MWCNTs was opened by oxidation with a nitric acid solution (65%) and refluxing them for 6 hrs as shown in Figure 1(b). Next, the treated MWCNTs were washed with distilled water many times to achieve the pH of 7.0 and dried at 90°C for overnight [19].

### 2.4. Preparation of MWCNT/ZnO Composites

The functionalized MWCNTs were dispersed in distilled water using an ultrasound bath for 2 hrs; then, 5 ml of ethylene glycol was added and blended for another 2.5 hrs at room temperature. Furthermore, 2.5 g of ZnO NPs was added with continued stirring and the temperature was raised to 80°C to dissolve the particles. Zn^+^ released by ZnO NPs was directly attracted to the carboxyl (–COOH) groups present on the surface of functionalized MWCNTs as shown in Figure 1. Finally, the mixture was annealed and dried at 80°C [20]. From here, four different composites (MWCNT/ZnO) with ZnO particles synthesized at different pH 6.0, 7.0, 8.0, and 10.0 were obtained.

### 2.5. Antibacterial Activity

The antibacterial activity of MWCNT/ZnO composites for ZnO NPs synthesized at pH 6.0, 7.0, 8.0, and 10.0 against *Staphylococcus aureus* (*S.A*), *Escherichia coli* (*E. coli*), *Klebsiella pneumonia* (*K.P*), and *Pseudomonas aeruginosa* (*Pseudo*) was studied by using agar well diffusion method [21]. The freshly grown cultures (media) of these bacteria were used as inoculums for antibacterial activity. 100 *μ*l of each MWCNT/ZnO composite was poured separately in wells (9 mm diameter) present on agar plates. The plates were then incubated in a thermal incubator at 40°C overnight. After the incubation period, the diameter of the zone of inhibition was measured in millimeters (mm).

### 2.6. Minimum Inhibitory Concentration (MIC) Assay

To investigate the MIC, the test was performed with standard protocols using 96-well plates [21]. A series of MWCNT/ZnO sample twofold dilutions were prepared across a corresponding row of a 96-well microtiter plate. For serial dilution, LB broth was used. A 106 CFU ml^−1^ cell density of *S.A*, *E. coli*, *K.P*, and *Pseudo* strains was mixed with an equal volume of broth. The microtiter plate was covered with an O_2_-permeable lid, incubated at 37°C. After overnight incubation, the minimal concentration of MWCNT/ZnO sample that prevented the clear suspension of 106 CFU ml^−1^ from becoming visibly turbid in the well was considered as the MIC. Each experiment was performed three times and repeated in a separate instant.

## 3. Result and Discussions

### 3.1. Morphological Analysis

The morphology of samples was studied by a field emission scanning electron microscope (FEI Nova NanoSEM 430). Figures 2(a) and 2(b) showed the micrographs of the pure MWCNT and functional multiwalled carbon nanotubes (FMWCNTs). The average diameter of MWCNT was 18 ± 4 nm. The FESEM images of multiwalled carbon nanotubes showed that the tubes were randomly and loosely entangled to each other, whereas in Figure 2(b), no effect on the structure of nanotubes took place by acid treatment during the process of functionalization. After the functionalization of MWCNT, the average diameter became 16 ± 3 nm, while the white spots appeared which suggested that the oxidation had taken place on the surface of FMWCNT. Figures 2(c)–2(f) show the micrographs of ZnO NPs prepared at pH 6.0, 7.0, 8.0, and 10.0, respectively. Large bulk particles with high agglomeration were observed in case pH 6.0 and 7.0. This agglomeration is a result of the acidic pH of the Zn(OH)_2_ solution during the synthesis process. Both samples lack sufficient OH^−^ ions [22].  Figure 2(e) shows that the ZnO nanoparticles are mostly rods in shape and are homogeneously distributed when the pH is increased to 8.0. When the pH is increased to pH 10.0, aligned flake microflowers/flakes accumulated with several sheets in one flower can be seen. The variation in morphology of zinc oxide NPs with pH was due to the ratio of H^+^ and OH^−^ in the solution during synthesis that controlled the hydrolysis and condensation of the solution [23]

(1) $$\begin{array}{c} \text{Zn}{\left(\text{Cl}\right)}_{2}+2\text{NaOH}⟶\text{Zn}{\left(\text{OH}\right)}_{2}+2\text{NaCl} \end{array}$$

(2) $$\begin{array}{c} \text{Zn}{\left(\text{OH}\right)}_{2}⟶{\text{Zn}}^{2+}+2{\text{OH}}^{-}⟶\text{ZnO}+{\text{H}}_{2}\text{O} \end{array}$$

(3) $$\begin{array}{c} \text{Zn}{\left(\text{OH}\right)}_{2}+{\text{OH}}^{-}⟶{\left[\text{Zn}{\left(\text{OH}\right)}_{4}\right]}^{2-} \end{array}$$

At low pH, more Zn^+2^ is formed (2) (deficiency of OH^−^) and results in agglomerated ZnO structures. When pH is increased to 8.0 or 10.0, the concentration of OH^−^ increases compared to Zn^+2^, and the [Zn(OH)_4_]^2-^ immediately starts to take place (3). The [Zn(OH)_4_]^2-^ acts as the new growth precursor; therefore, anisotropic growth of ZnO occurred at the active site of the ZnO seed. Similarly, Figures 2(g)–2(j) show the micrographs of MWCNT/ZnO for ZnO synthesized at pH 6.0, 7.0, 8.0, and 10.0. The surface of MWCNTs/ZnO shows that MWCNTs form a mesh-like structure in which ZnO NPs are embedded on the surface of MWCNTs and form the bond with functional groups on the surface of functionalized MWCNT. In conclusion, the composite structures have a well-dispersed carbon nanotube network.

Furthermore, the properties of ZnO NPs and MMWCNTs/ZnO were explored using energy-dispersive X-ray (EDX) which identifies the elements in the sample. Figures 2(h)–2(j) show the EDX spectra of ZnO NPs synthesized at pH 10.0. The spectra confirmed the existence of both zinc and oxygen as shown in Table 1. EDX spectra revealed the presence of Cl in FMWCNT and MWCNT/ZnO composites. The EDX analysis also indicates that the Cl component is more in FMCNTs compared to composites which shows some residues are left during washing of MWCNTs with HCl and these residues are suppressed when the solution pH is changed to 10.0. However, it can be seen in Table 1 that the weight percentage of C increased as the MWCNTs form composites with ZnO NPs. The results confirm that the sample contains Zn, O, and carbon as well as confirm the formation of MWCNTs/ZnO.

### 3.2. Structural Analysis

The crystalline phase of prepared ZnO NPs at different pH 6.0, 7.0, 8.0, and 10.0 and their composites were analyzed with XRD. The XRD pattern of MWCNT and FMWCNT is shown in Figure 3(a). In Figure 3(a), the peaks (002), (100), and (110) are indexed for pure MWCNT which are found at 26°, 43°,_,_ and 77° [24]. The XRD patterns of the pure and functionalized MWCNT show similar peaks, but MWCNT spectra are slightly less strong than FMWCNT. The diffraction peaks (002), (100), and (110) corresponding to the functionalized multiwalled carbon nanotubes became evident around 26°, 43°, and 77° and showed that the structure of the functionalized MWCNTs has not been destroyed after the acid treatment process.

Figure 3(b) shows the XRD pattern of ZnO NPs prepared at pH values of 6.0, 7.0, 8.0, and 10.0. The samples prepared at pH 6.0 showed no definite peaks of pure ZnO. It is observed that the ZnO structure has not been well synthesized at pH 6.0. This was due to the of a high concentration of H^+^ ions and a low concentration of OH^−^ ions in the solution. However, at pH 7.0, ZnO peaks are obtained but peaks are broader and less intense. However, ZnO NPs withpH ≥ 8showed the crystalline nature with all peaks (100), (002), (101), (102), (110), (103), (200), (112), (201), and (202) which are found to be at position 31.67°, 34.31°, 36.14°, 47.40°, 56.52°, 62.73°, 66.28°, 67.91°, 69.03°, and 77.03°, respectively [25]. It can be observed that the peak intensity of (101) increased as pH changed from 5.0 to 10.0. This intense peak at high pH revealed that ZnO NPs had no impurity and represents the hexagonal wurtzite structure. The lattice parameters (*a* = *b* = 3.25 Å and *c* = 5.20 Å) for ZnO NPs were measured for the peaks that confirm the hexagonal wurtzite structure as confirmed by the JCPDS 36-1451 data. ForpH ≥ 7, the ZnO peaks were observed which shows that the precursors were completely decomposed and no other products were formed. Additionally, higher intensity and narrower width peaks confirmed that the obtained ZnO NPs have good crystallinity for pH ≥ 8.

Figure 3(c) shows the XRD pattern of MWCNT/ZnO for pH values 6.0, 7.0, 8.0, and 10.0. Similar to ZnO NPs at pH 6.0, the MWCNT/ZnO at pH 6.0 shows no definite peak of ZnO NPs, but the peak (002) at 26° appears which shows the presence of MWCNTs in agglomerated ZnO NPs. However, the same composite MWCNTs/ZnO for at pH 7.0, 8.0, and 10.0 were well synthesized. Moreover, it is observed that the peaks of zinc oxide are dominated over the peaks of MWCNT due to zinc oxide present on the surface of MWCNT. It was found that MWCNT and ZnO NPs were crystallized with hexagonal phase.

### 3.3. Fourier Transform Infrared Spectroscopy (FTIR) Analysis

FTIR was performed to analyze the presence of functional groups and the quality of synthesized materials. The spectrum was plotted in the range of 500–4000 cm^−1^. The FTIR spectrum of MWCNT, FMWCNT, ZnO NPs, and MWCNT/ZnO composites synthesized at pH 6.0, 7.0, 8.0, and 10.0 is shown in Figures 4(a)–4(c).  Figure 4(a) shows the FTIR spectra of MWCNT, and peaks at 1274 cm^−1^ and 1714 cm^−1^ were attributed to the carboxylic group bands C-O and C=O, respectively. The peak at 3449 cm^−1^ confirmed the presence of hydroxyl group –OH, whereas in FMWCNTS, carboxylic groups formed on the surface of MWCNT by acid treatment are shown at 1800 cm^−1^ and stretching at about 3466 cm^−1^ [26]. Similarly, FTIR spectra of ZnO NPs are shown in Figure 4(b). The peak at 3448 cm^−1^ showed the presence of the –OH group. From the figure, it can be observed that the position of –OH peak changes from pH 6.0 to a broad peak at pH 10.0. This moment of –OH peak plays an important role in the formation of ZnO NPs, which can be seen in FESEM images, while the C-O-C peak is appearing between 1025 and 943 cm^−1^ and the peak at 2360 cm^−1^ showed the presence of C=O. The peaks of C=O and C-O-C are not much affected on the synthesis of ZnO NPs as the bands are not much different with pH change. The ZnO absorption band near 529 cm^−1^ was observed in the spectrum of ZnO NPs. From the graph, it can be observed that all peaks of ZnO were shifted due to changes in the morphology of ZnO NPs. In a similar manner, Figure 4(c) shows the FTIR spectra of MWCNT/ZnO. In MWCNT/ZnO NPs, the peak at 3402 cm^−1^ corresponded to the –OH vibrational mode which appears due to the possible water and acid used during the purification process identified from the MWCNT sample [27]. The peak at 1210 and 1553 cm^−1^ is related to the C-H and C=C band characteristics of carbon nanotubes [28]. The peak at 552 cm^−1^ and 977 cm^−1^ is related to the characteristics for ZnO and Zn-C for MWCNTs/ZnO, providing the MWCNT decoration with ZnO NPs [29, 30].

### 3.4. Thermal Analysis of ZnO and ZnO/MWCNTs

TGA is a useful method of thermal analysis based on the measurement of mass change related to the temperature for the quantitative determination of the thermal degradation. The thermal properties of ZnO NPs were determined by TGA/DSC (Mettler Toledo TGA/DSC 1). The ZnO NPs (not annealed or as-synthesized) were heated up to 800°C at 10°C/min. The results obtained are shown in Figure 5(a). There are two major losses in the raw ZnO NPs. The first mass loss ~100°C can be seen due to the removal of water, while the second mass loss near 250°C is the removal of byproducts (unreacted products in the reaction). In the next step, the TGA/DSC has performed again for the annealed sample. The TGA/DSC results of annealed ZnO NPs are shown in Figure 5(b). The melting point of pure ZnO is ~1970°C, that is why pure zinc oxide is very stable up to very high temperatures, which can be seen in Figure 5(b), the material showing perfect thermal stability up to 800°C [31].  Figure 5(c) shows the TGA/DSC of pure MWCNTs. It shows one major loss which may be attributed to the gasification of MWCNTs at which its decomposition begins at 550°C [32]. As it can be seen, the mass loss of ZnO NPs is slight, whereas the thermal degradation of MWCNTs is large. The TGG/DSC analysis of MWCNT/ZnO with ZnO NPs synthesized at different pH = 6.0, 7.0, 8.0, and 10.0 is shown in Figures 5(d) and 5(e). It can be seen that the composite synthesized at pH = 6.0 and 7.0 is less stable compared to pH = 8.0, 10.0, whereas from Figure 5(e) (DSC curve), it can be seen that there are two endothermic peaks at 133 and 650°C, respectively. The endothermic peak at 133°C might stem from the loss of crystalloid water and that at 650°C, it could be due to the presence of residue [33].

## 4. Antibacterial Activity

### 4.1. Qualitative Antimicrobial Assay

Bacterial resistance is based on its defensive barriers which are the cell wall and cell membrane. Nanoparticles (NPs) use different pathways of cell membranes to adsorb in gram-positive and gram-negative bacteria [34]. For antibacterial activity, the NPs came in contact with bacterial cell wall by electrostatic attraction, van der Waals forces, receptor-ligand, and hydrophobic interactions to cross the membrane [35]. All these will affect the metabolic activities of bacteria and cause the deactivation of protein by interacting with enzymes, ribosomes, and DNA as mechanism shown in Figure 6(a). The ZnO NPs create zinc ions which generate reactive oxygen species (ROS). As a result, it not only causes oxidative stress but also alters the cell membrane permeability, unbalancing the electrolyte, inhibiting the enzyme, and deactivating protein [36]. The antibacterial activity of MWCNT/ZnO composites for ZnO NPs synthesized at pH 6.0, 7.0, 8.0, and 10.0 was examined against *Staphylococcus aureus* (*S.A*), *Escherichia coli* (*E. coli*), *Klebsiella pneumonia* (*K.P*), and *Pseudomonas aeruginosa* (*Pseudo*) as shown in Figures 6(b)and 6(c). The MWCNT/ZnO composites for ZnO NPs synthesized at pH 7.0, 8.0, and 10.0 show better results compared to MWCNT/ZnO composites for ZnO NPs synthesized at pH 6.0, respectively. It can be observed that *S.A* bacteria were more sensitive compared to *E. coli*, *K.P*, and *Pseudo* for MWCNT/ZnO composites. The observed value of the zone of inhibition is shown in Table 2. The different responses towards antibacterial activity were observed for MWCNT/ZnO composites. At pH 6.0 or 7.0, the ZnO NPs are in the form of agglomerated or bulk NPs. As pH increased to 10.0, the shapes changed from rod to flakes/microflowers. The antibacterial activity is strongly dependent on the shape and size of NPs. The MWCNT/ZnO NPs synthesized at pH 6.0, 7.0, 8.0, and 10.0 change the morphology of ZnO NPs which reduces the particle size thereby increasing the attachment of composite to the bacteria and damaging the cell membrane integrity. Based on the antibacterial activity results, the MWCNTs/ZnO NPs synthesized at pH 10.0 show a significant zone of inhibition for all types of bacteria. The increased antimicrobial activity occurs due to the presence of the NPs and FMWCNTs. When functional groups are introduced on the surface of MWCNTs, it results in an increase in the dispersion of ZnO/MWCNTS composites. Therefore, the MWCNT surface modified with NPs and the functional group can form stable dispersion which affects the interaction with spore disrupting cell membrane integrity, reducing cell surface hydrophobicity, and downregulating the transcription of oxidative stress-resistance genes in bacteria. In the present research, the strongest antibacterial activity was observed for *S.A*. These results suggest that the efficiency is limited against gram-negative bacteria. This can be related to the particularities of their cellular wall (single-layered structure) and eukaryote organization.

### 4.2. Minimum Inhibitory Concentration (MIC) Assay

Quantitative tests suggested that MWCNTs/ZnO NPs synthesized at pH 10.0 have more pronounced antibacterial effects compared to other composite (Figure 7). The values of the MIC were also influenced by the microbial strain tested. In the case of MWCNT/ZnO NPs synthesized at pH 10.0, the MIC values obtained for *S.A*, *E. coli*, *K.P*, and *Pseudo* were 0.25%, 0.5%, 0.5%, and 1%, respectively. This showed that MWCNT/ZnO NPs synthesized at pH 10.0 are most effective against S.A, where they successfully inhibit the growth of bacteria at the MIC as low as 0.25 mgml^−1^.

## 5. Conclusion

In the present work, novel composite MWCNT/ZnO NPs synthesized at different pH 6.0, 7.0, 8.0, and 10.0 are reported to improve the antibacterial activity. The formation of MWCNT/ZnO composites was confirmed by morphological, structural, and FTIR analysis. The variation of pH showed different morphologies from agglomerated structures to rod-like than flower-like structures. The in vitro results of MWCNT/ZnO composites show significant antibacterial activity against S.A, E. coli, K.P, and Pseudo strains. The higher antibacterial activity was observed for S.A with the largest diameter of zone of inhibition (20 mm). These results suggest that MWCNT/ZnO has potential application as an antibacterial material for simultaneous concentrating and inactivating pathogenic bacteria.

## Figures and Tables

**Figure 1:** Schematics for the synthesis of MWCNT/ZnO composite.

**Figure 2:** FESEM micrograph of (a) MWCNT, (b) FMWCNT, (c-f) ZnO NPs, (g–j) ZnO NPs at magnification of 1 *μ*m, and (k–n) MWCNT/ZnO composites with ZnO synthesized at pH 6.0, 7.0, 8.0, and 10.0. (o–q) EDX pattern of MWCNT, ZnO NPs, and MWCNT/ZnO at pH 10.0, respectively.

**Figure 3:** The X-ray diffraction pattern of (a) MWCNT and FMWCNTs, (b) ZnO NPs, and (c) MWCNT/ZnO composites with ZnO NPs synthesized at pH = 6.0, 7.0, 8.0, and 10.0.

**Figure 4:** Fourier transform infrared radiation spectrum of (a) MWCNT and FMWCNT, (b) ZnO NPs, and (c) MWCNT/ZnO with ZnO NPs synthesized at pH = 6.0, 7.0, 8.0, and 10.0, respectively.

**Figure 5:** Thermograms showing the mass loss of the (a) ZnO as grown, (b) ZnO annealed, (c) MWCNTs, and (d, e) the MWCNT/ZnO composites with ZnO NPs synthesized at pH = 6.0, 7.0, 8.0, and 10.0.

**Figure 6:** (a) Mechanism for antibacterial activity of MWCNT/ZnO composite. (b) Zone of inhibition attained by MWCNT/ZnO composites against bacteria *Staphylococcus aureus* (*S.A*), *Escherichia coli* (*E. coli*), *Klebsiella pneumonia* (*K.P*), and *Pseudomonas aeruginosa* (*Pseudo*) strains. (c) Graphical representation of zone of inhibition attained by MWCNT/ZnO composites against the bacterial strain.

**Figure 7:** MIC representation of MWCNTs on bacterial strains tested at 37°C for overnight incubation. Data represented were mean of triplicate values with standard deviation.

**Table 1:** Elemental analysis by EDX of MWCNT/ZnO composites with synthesized ZnO NPs at different pH values.

Elements	MWCNTs	ZnO (pH = 10.0)	MWCNTs/ZnO
	Weight%	Weight%	Weight%
Zn	—	66.5	79.3
O	—	21.4	13.0
C	89.3	—	7.6
Cl	—	12.1	0.1

**Table 2:** Comparison of antibacterial activity of MWCNT/ZnO composites synthesized at different pH.

Organisms	pH 6.0 (1) (mm)	pH 7.0 (2) (mm)	pH 8.0 (3) (mm)	pH 10.0 (4) (mm)
(a) Staphylococcus aureus (S.A)	16	18	19	20
(b) Escherichia coli (E. coli)	14	14	18	19
(c) Klebsiella pneumonia (K.P)	11	16	18	18
(d) Pseudomonas aeruginosa (Pseudo)	10	12	17	18

∗Included “9 mm” well size.

## Data Availability

The data that support the findings of this study are available from the corresponding author upon reasonable request.
